This article has been retracted.

# Dihydromyricetin Attenuates Inflammation through TLR4/NF-kappaB Pathway

**DOI:** 10.1515/med-2019-0083

**Published:** 2019-09-15

**Authors:** Nianshui Jing, Xinnan Li

**Affiliations:** 1 Department of Pharmacy, Jinan No.2 People’s Hospital, Jingyi Road 148, Jinan 250001, Shandong, China

**Keywords:** Dihydromyricetin, inflammation, TRL4, NF-κB

## Abstract

Microglia plays a complex role in neuroinflammation, which has been implicated in neurodegenerative diseases such as Alzheimer’s disease and Parkinson’s disease. This study aims to explore the effect and mechanism of Dihydromyricetin (DHM) on lipopolysaccharide (LPS)-induced inflammation in microglial BV-2 cells. Cell viability was measured by 3-[4,5-dimethylthiazol-2-yl]2,5-diphenyltetrazolium bromide (MTT) assay. The pro-inflammatory mediators and cytokines including interleukin (IL)-6, IL-1β, and tumor necrosis factor-α (TNF-α); inducible nitric oxide synthase (iNOS); and cyclooxygenase 2 (COX-2) were measured by enzyme-linked immunosorbent assay (ELISA) and/or quantitative real-time PCR (qRT-PCR). The expression of p-p65, p-IκBα, toll-like receptor 4 (TLR4), and myeloid differentiation primary response 88 (MyD88) were analyzed by western blot. The present study showed that DHM treatment alleviated LPS-induced viability reduction, suppressed the mRNA levels of IL-6, IL‐1β and TNF-α, inhibited the mRNA and protein expression of iNOS and COX-2, and attenuated the activation of NF-кB and TLR4 signaling in a concentration-dependent manner. In conclusion, DHM exerts an anti-inflammatory effect on LPS-induced BV-2 microglial cells, possibly through TRL4/NF-κB signaling pathway.

## 1 Introduction

The age-related neurodegenerative disorders such as Alzheimer’s disease (AD), Parkinson’s disease (PD), Huntington’s disease (HD), amyotrophic lateral sclerosis (ALS) and stroke are characterized by the excessive neuroinflammatory responses in the central nervous system (CNS) [1, 2, 3, 4]. Microglial cells, the major resident macrophages in the CNS parenchyma, serve as the first line of host defense and protect the CNS from insults [5]. The quiescent microglia cells are ramified. Once activated by microbial infection, pathological stimuli or brain injuries, microglial cells may change into an amoeboid morphology and secrete pro-inflammatory cytokines (e.g. TNF-α, IL-1β and IL-6), ultimately leading to clinically significant neuronal damage or death and dysfunction in the CNS [6, 7]. Thus, the suppression of activated microglia and the protection of neurons from neuroinflammation have been suggested to be a potentially promising strategy for the prevention and treatment of neurodegenerative disorders.

Natural compounds from herbs are one of the important sources for development of new drugs [8]. Dihydromyricetin (DHM; C_15_H_12_O_8_) is a natural flavanol compound isolated from *Ampelopsis grossedentata*, a traditional Chinese medicine that is reported to have multiple pharmacological activities including anti-oxidative, anti-cancer and anti-alcohol in toxication [9]. Previous studies have shown that DHM ameliorates behavioral deficits and reverses neuropathology in the transgenic mouse models of AD and PD. Moreover, DHM has been demonstrated to exhibit anti-inflammatory effects, as evidenced by suppressing the expressions of TNF-α and IL-6 mRNA. However, the mechanism of its anti-inflammatory effects has not been fully investigated.

In the present study, we aimed to explore the effect and mechanism of DHM on lipopolysaccharide (LPS)-induced inflammation in microglial BV-2 cells.

## 2 Methods

### 2.1 Chemicals

DHM (purity>98%) was purchased from the Lyphar Biotech Co., Ltd (Xi’an, China) and dissolved in dimethyl sulfoxide (DMSO, <0.05%, v/v, without detectable effects) for all study experiments.

### 2.2 Cell culture

The immortalized murine microglial cell line BV-2 was purchased from the Chinese Academy of Medical Sciences (Beijing, China). BV2 cells were cultured in Dulbecco’s Modified Eagle’s Medium (DMEM, HyClone Inc., UT, USA) supplemented with 10% fetal bovine serum (HyClone Inc., UT, USA), penicillin (100 U/mL) and streptomycin (100 U/ mL) in a humidified incubator containing 95% air and 5% CO_2_ at 37°C.

### 2.3 MTT assay

Cell viability was determined by the MTT method following the manufacturer’s instructions. Briefly, microglial BV-2 cells were seeded in 96-well plates at a density of 2×10^4^ cells/well and cultured with LPS (0.1 μg/mL) and/ or various concentrations of DHM (20, 40, 80 or 100 mg/L) for 48h. After incubation, 20 μl/well of 3-[4,5-dimethylthiazol-2-yl]2,5-diphenyltetrazolium bromide (MTT) solution (Sigma-Aldrich, USA) was added to each well, and then cells were incubated for an additional 4 hour. Plates were then centrifuged to remove the supernatants, and the crystals were dissolved in 150 μL of DMSO. The spectrophotometrical absorbance of the samples was measured using a quantified microplate reader at a wavelength of 490 nm. Each assay was performed in triplicates.

### 2.4 ELISA assay

After obtaining cell supernatants, the concentrations of IL‐6, IL‐1β and TNF-α were measured using enzyme-linked immunosorbent assay (ELISA) kits (Chenglin Biotechnology, Beijing, China) according to the manufacturer’s instructions. Each assay was performed in triplicates.

### 2.5 Real-time PCR

Total RNA was isolated from BV-2 cells using RNAiso Plus Reagent (Takara, Dalian, PR China), and reverse-transcribed by using PrimeScript^TM^RT Reagent Kit (Takara, Dalian, China) to produce cDNA. The quantitative real-time PCR (qRT-PCR) was performed with SYBR^®^ Premix Ex Taq™ (Tli RNase Plus) (Takara, Dalian, china). Glyceraldehydes-3-phosphate dehydrogenase (GAPDH) mRNA was used as an internal control. The quantitative PCR program used was as follows: predenaturation (95°C, 5 min), denaturation (95°C, 20 sec), annealing (55°C, 20 sec), and extension (72°C, 45 sec), using primers specific for iNOS, COX-2, IL-6, IL‐1β and TNF-α.

### 2.6 Western Blotting

BV-2 microglial cells were lysed with radioimmunoprecipitation assay buffer (Beyotime Biotechnology, Shanghai, China) supplemented with protease inhibitors (Roche, Basel, Switzerland); 30 μg samples of the lysates were separated on 12% SDS-PAGE gels and transferred to polyvinylidene fluoride membranes. The membranes were incubated with primary antibodies overnight at 4°C. The primary antibody incubation was followed by incubation with horseradish peroxidase-conjugated secondary antibodies. The bound antibodies were detected using an ECL kit (ComWin Biotech Co., Beijing, China). Primary antibodies were as follows: p-p65 (Santa Cruz Biotechnology, Santa Cruz, CA, USA; 1:1000), p-IкBα (Abcam; 1:500), TLR4 (Santa Cruz; 1:1000), myeloid differentiation primary response 88 (MyD88; Santa Cruz; 1:1000) and β-actin (Santa Cruz; 1:1000). β-actin was used as a loading control.

### 2.7 Statistical analysis

All quantitative data were expressed as mean ± standard deviation (SD) and compared by the Student’s t-test and one-way Analysis of Variance (ANOVA) followed by Turkey’s *post-hoc* analysis. Chi-square test and Fisher’s exact test were used to compare categorical variables. All tests were 2-sided and a *P* value<0.05 was considered significant.

All statistical analyses were performed with the SPSS statistical software program package (SPSS version 20.0 for Windows, SPSS Inc., Chicago, Illinois, USA).

## 3 Results

### 3.1 DHM attenuated LPS-induced viability reduction in microglial BV-2 cells

The viability of BV-2 microglia under LPS and various concentrations of DHM were evaluated using the MTT assay. As shown in Figure 1a, there was no significant difference in the cell viability between the control group and various doses of DHM (*P*>0.05), indicating that DHM did not exhibit cytotoxicity on BV-2 cells. The viability of BV-2 cells was significantly reduced in the presence of LPS simulation (*P*<0.01), and treatment with various doses of DHM all improved LPS-induced viability reduction (all *P*<0.01, Figure 1b).

**Figure 1:** The effects of various concentrations of DHM (20, 40, 80 or 100mg/L) on the viability of BV-2 microglial cells using the MTT assay. (a) DHM did not exhibit cytotoxicity on BV-2 microglial cells; (b) DHM (20, 40, 80 or 100mg/L) significantly suppressed the LPS-induced viability reduction of BV-2 microglial cells. *P<0.01 compared with control group; #P<0.01 compared with LPS group.

### 3.2 DHM attenuated LPS-induced inflammatory responses in microglial BV-2 cells

The pro-inflammatory cytokines IL-6, IL‐1β and TNF-α were measured by ELISA to evaluate the effect of DHM on LPS-induced inflammatory responses. As shown in Figure 2a-c, LPS significantly induced the release of IL-6, IL‐1β and TNF-α (*P*<0.01). Following the treatment with various doses of DHM, the up-regulation of all these pro-inflammatory cytokines was attenuated (*P*<0.01). In addition, the mRNA levels of IL-6, IL‐1β and TNF-α were measured by qRT-PCR. The results illustrated in the Figure 2d-f showed that LPS-induced overproduction of IL-6, IL‐1β and TNF-α mRNA was inhibited by DHM (*P*<0.01). It is observed that the reductions in secretion levels and mRNA levels of pro-inflammatory cytokines were significantly greater in LPS-induced microglial BV-2 cells treated with 80 and 100 mg/L of DHM, compared with those with 20 and 40 mg/L of DHM (*P*<0.01). These results suggested that DHM could attenuate LPS-induced inflammatory responses in a dose-dependent manner.

**Figure 2:** The effects of various concentrations of DHM (20, 40, 80 or 100mg/L) on inflammatory response. (a-c) DHM (20, 40, 80 or 100mg/L) significantly suppressed the LPS-induced upregulation of pro-inflammatory cytokines IL-6, IL‐1β and TNF-α in BV-2 microglial cells. (d-f) DHM (20, 40, 80 or 100mg/L) significantly suppressed the LPS-induced increased mRNA levels of IL-6, IL‐1β and TNF-α in BV-2 microglial cells. *P<0.01 compared with control group; ^#^P<0.01 compared with LPS group; ^Δ^P<0.01 compared with DHM 20 or 40 mg/L groups.

### 3.3 DHM attenuated LPS-induced elevated mRNA expression of iNOS and COX-2 in microglial BV-2 cells

iNOS and COX-2 have been regarded as two important bio-markers of inflammatory response, whose mRNA expressions were evaluated by qRT-PCR. It is shown that the mRNA expressions of iNOS (Figure 3a) and COX-2 (Figure 3b) were significantly increased after simulated by LPS (*P*<0.01), while DHM could significantly attenuated the upregulated mRNA in a dose-dependent manner. The mRNA expressions of iNOS and COX-2 were significantly lower in the LPS-induced microglial BV-2 cells treated with 80 and 100 mg/L of DHM, compared with those with 20 and 40 mg/L of DHM (*P*<0.01).

**Figure 3:** The effects of various concentrations of DHM (20, 40, 80 or 100mg/L) on mRNA levels of nitric oxide synthase (iNOS) and cyclooxygenase 2 (COX-2). (a) DHM (20, 40, 80 or 100mg/L) significantly suppressed the LPS-induced increased mRNA level of iNOS. (b) DHM (20, 40, 80 or 100mg/L) significantly suppressed the LPS-induced increased mRNA level of COX-2. *P<0.01 compared with control group; ^#^P<0.01 compared with LPS group; ^Δ^P<0.01 compared with DHM 20 or 40 mg/L groups.

### 3.4 DHM attenuated LPS-induced activation of NF-кB and TLR4 signaling

TLR4 medicated signaling predominately actives NF-κB that plays a vital role in the expression regulation of groups of genes involved in immune and inflammatory responses as well as neuroinflammation-associated disease pathogenesis [10, 11]. As shown in Figure 4a-c, the expressions of p-p65 and p-IкBα were significantly increased by the LPS simulation, and DHM treatment effectively inhibited their expressions in a concentration-dependent manner, indicating that DHM inhibited the LPS-induced activation of NF-кB pathway. Meanwhile, the expressions of TLR4 and MyD88 were significantly increased in LPS-induced microglia, which were attenuated by DHM in a dose-dependent manner (Figure 4d-f). It is found that the mRNA expressions of p-p65, p-IкBα, iNOS and COX-2 were significantly lower in the LPS-induced microglial BV-2 cells treated with 80 and 100 mg/L of DHM, compared with those with 20 and 40 mg/L of DHM (*P*<0.01). Thus, the LPS-induced inflammatory response may be attenuated by DHM through inhibiting the TLR4/NF-кB signaling pathway.

**Figure 4:** The effects of various concentrations of DHM (20, 40, 80 or 100mg/L) on NF-κB and toll-like receptor 4 (TLR4) signaling. (a-c) The activation of NF-κB induced by LPS was attenuated by DHM (20, 40, 80 or 100mg/L). (d-f) The activation of TLR4 signaling induced by LPS was attenuated by DHM (20, 40, 80 or 100mg/L). *P<0.01 compared with control group; ^#^P<0.01 compared with LPS group; ^Δ^P<0.01 compared with DHM 20 or 40 mg/L groups.

## 4 Discussion

A large amount of studies have demonstrated the crucial role of neuroinflammation with excessively activated microglia in the pathology of neurodegenerative diseases. The present study showed that DHM treatment alleviated LPS-induced neurotoxicity, suppressed the inflammatory responses, inhibited the secretion of iNOS and COX-2, and attenuated the activation of NF-кB and TLR4 signaling.

The persistent and uncontrolled activated microglial cells is an important feature of neurodegenesrative diseases. Over-activation of microglia releases pro-inflammatory cytokines including IL-6, IL‐1β and TNF-α, which would lead to the damage of neurons and further active the inflammatory cascade [12]. It is reported that IL-6, IL‐1β and TNF-α are significantly elevated in patients with AD [13] and PD [14]. In addition, the activated microglial cells also produce harmful substances, such as iNOS, COX-2 and other free radicals, which may perturb neuronal death and induce the development of neurodegeneration [15]. Our study showed that DHM significantly inhibited the iNOS and COX-2 expressions and also down-regulated the expression of pro-inflammatory cytokines, indicating that DHM suppressed the inflammatory responses in microglia and may thus be beneficial in the treatment of neurodegenerative disorders.

The transcription factor NF-kB plays a crucial role in the innate inflammatory response and is a key mediator that is responsible for several critical biological processes such as immune and inflammatory responses. The activation of NF-kB is triggered in the microglia upon stimulation [16], which will regulate the inflammatory pathway by stimulating the secretion of ROS and pro-inflammatory cytokines such as IL-6, IL‐1β and TNF-α and thus play secondary neurotoxicity effects [17]. Notably, NF-kB expression is highly elevated in brain samples from PD patients [18]. In the present study, DHM is demonstrated to attenuate the elevated expressions of p-p65 and p-IкBα, indicating that the NF-kB activation was inhibited by DHM.

Toll-like receptors (TLRs) are first-line molecules for initiating innate immune responses. Among more than ten mammalian TLRs identified [19], TLR4 has been shown to be expressed on microglia and mediates neuroinflamma-tory diseases [20]. Furthermore, MyD88, a critical adapter protein for TLR4, leads to the activation of downstream NF-𝜅B and the subsequent production of pro-inflammatory cytokines implicated in neurotoxicity [21]. Recently, Zhou et al. reported that TLR4/NF-𝜅B/cytokines signaling is obviously activated in MPP-induced BV-2 cells. They concluded that TLR4 signaling displays a critical role in the activation of BV-2 cells in response to inflammatory response [22]. Our study showed that DHM attenuated LPS-induced TLR4 signaling.

In conclusion, our study indicated that DHM exerts an anti-inflammatory effect on LPS-induced BV-2 microglial cells, possibly through TRL4/NF-kB signaling pathway.
